The article "International Trade of Masks and COVID-19 Pandemic Containment" was published in 2022. Journal: J Environ Public Health.

# International Trade of Masks and COVID-19 Pandemic Containment

**DOI:** 10.1155/2022/2156950

**Published:** 2022-07-09

**Authors:** Xiayang Fan, Bing Li, Yuanyuan Xiu

**Affiliations:** ^1^School of International Trade and Economics, Central University of Finance and Economics, Beijing 102206, China; ^2^Lingnan College, Sun Yat-sen University, Guangzhou 510275, China; ^3^School of Business, Beijing Union University, Beijing 100101, China

## Abstract

This study analyzes the impact of the exports of China's masks and other antivirus supplies on the people from the importing countries who are subject to the severe pandemic during the coronavirus disease 2019 (COVID-19) pandemic. Our main data include the COVID-19 cases data of countries around the world published by Johns Hopkins University and the data of China's exports of masks or other antivirus supplies to these countries from the Chinese Customs Database. Using cross-sectional data of about 180 countries and multiple regression analysis, we find that the antivirus supplies from China have played an important role in combating the COVID-19 pandemic. Specifically, China's masks are shipped to countries around the world, and these masks can improve the recovery rate and protect people against the COVID-19 pandemic. Our findings are relevant to global efforts in the COVID-19 pandemic containment.

## 1. Introduction

At the end of 2019, a group of patients with unexplained form of viral pneumonia flooded into the hospital. This announced a large-scale outbreak of pneumonia with unknown origin, and the medical system in Wuhan, China, was facing a huge challenge for a time. On February 11, 2020, the World Health Organization (WHO) officially named the new coronavirus COVID-19 [1]. On March 11, 2020, the WHO announced that the COVID-19 virus was officially a pandemic after barreling through 114 countries and infecting over 118,000 people [2]. It can be seen that the virus spread quickly, causing a severe situation. Until the end of 2021, in the globalized world, the virus has infected nearly 320,000,000 people, causing over 5,000,000 deaths and more than 200 countries and regions are affected by it.  Figure 1 shows the rapid deterioration of the situation in countries other than China from February 2020 to July 2021. However, the COVID-19 pandemic is far from over.

As the first country in the world to have a large-scale outbreak of the COVID-19 pandemic, China has taken various measures as soon as possible, such as locking down Wuhan, prohibiting the mobility of people in various regions, and providing emergency support to Wuhan. Wuhan was locked on January 23, 2020, and all traffic channels were closed to prevent the spread of the virus. After the pandemic was effectively controlled, Wuhan's lockdown was lifted on April 8, 2020, and this indicated a temporary victory for China in fighting the terrible pandemic. However, the pandemic was still wildly prevalent in the rest of the world. Due to the spread of the pandemic, production in most countries around the world has been hampered. China is the factory of the world and is connected to the world through international trade. After the global outbreak of the pandemic, China took the lead in resuming work and production. China's export of antivirus supplies continues to increase.

Even before the COVID-19 pandemic broke out, China's exports of antivirus supplies, especially masks, accounted for a large proportion of global market. We use the data of bilateral trade flows in the BACI database (https://www.cepii.fr/cepii/en/bdd_modele/presentation.asp?id=37) and the antivirus supplies introduced in Section 3.1.2 to draw Figure 2. It shows the absolute quantity and the relative proportion of China's exports of antivirus supplies and the total global exports from 2012 to 2019; Obviously, China's exports of total antivirus supplies, final goods, and intermediate goods (Section 3.1.2 for the selection and classification of antivirus supplies.) account for more than 20% of the world's exports. It is worth noting that the export of masks accounts for about 60% of the world's total exports.

Since the pandemic situation in China was well controlled in April 2020, according to the statistics of the General Administration of Customs of China (https://www.customs.gov.cn/customs/xwfb34/mtjj35/3045505/index.html), the average daily exports of major antivirus supplies in China have increased from 1 billion yuan in early April to 2 billion yuan in the middle period and then to more than 2.5 billion yuan in May. From Figure 3(a), it can be seen that in April 2020, the export value of China's antivirus supplies has greatly increased; Figure 3(b) shows that the value and weight of masks exported by China have greatly increased.

According to our knowledge, there are no such studies about the impact of China's export of masks and antivirus supplies on fighting against the pandemic in countries around the world. However, exploring this relationship is important for pandemic containment. Meanwhile, at the beginning of the new year, President Xi Jinping mentioned in his 2022 New Year's message (https://baijiahao.baidu.com/s?id=1720660035235352908&wfr=spider&for=pc) “When I communicated with foreign leaders and heads of international organizations by telephone and video, they repeatedly praised China's efforts to fight the pandemic and its contribution to the prevention and control of the global pandemic.” However, there is no systematic evidence to verify this argument yet. This study tries to provide some statistical tests for that and enriches literature related to China's contribution to the fight against the pandemic. In addition, this study complements the literature on international trade and the spread of virus with new perspectives.

Our findings support the significant role of masks in fighting against the COVID-19 pandemic. During the pandemic, China's exports of masks have contributed to a rise in recovery rates in the importing countries affected by the COVID-19 pandemic. Compared with the previous research, which believes that international trade promotes the spread of the virus, the results of the study show that when the traded products are antipandemic supplies, it will be conducive to the containment of the pandemic.

There are two main research objectives in this study. The first is to find the relationship between China's export of masks and antivirus supplies and global pandemic containment. The second is to explore the role of collectivism in this relationship. Based on the above goals, the remainder of the study proceeds as follows.  Section 2 provides a literature review.  Section 3 describes our data and empirical strategy.  Section 4 presents the benchmark results, heterogeneous effects, mechanism analysis, robustness checks, and discussion.  Section 5 concludes with a discussion of the implications of these results for both future research on COVID-19 pandemic containment.

## 2. Literature Review

The existing research on the COVID-19 pandemic is mainly divided into two categories. The first part is to study the characteristics of the virus and its serious harm to public health. The second part is to study the containment of the COVID-19 pandemic, including the importance of wearing masks in stopping the spread of the pandemic, China's efforts in fighting the COVID-19 pandemic, and the relationship between international trade and the spread of infectious diseases.

### 2.1. The Harm of the COVID-19 Pandemic

The COVID-19 pandemic spreads rapidly by human-to-human transmission [3]. COVID-19 is spread primarily via respiratory droplets—little blobs of liquid released as someone coughs, sneezes, or talks. Viruses contained in these droplets can infect other people via eyes, nose, or mouth—either directly landing on someone's face or being transferred there by people touching their faces with contaminated hands [4,5]. At the same time, the virus poses a great threat to people's lives and health. It is mainly manifested as fever, fatigue, dry cough, and so on. Most patients have a good prognosis, while a few patients are in critical condition and even die [3,6].

It is worth noting that COVID-19 virus has not only brought great harm to people's health but also caused “panic shortage of medical resources.” The speed of regional expansion and the sudden increase in the number of cases shocked the health and public health services in China, especially in Wuhan and Hubei, and quickly became overwhelmed [7]. Moreover, the pandemic not only crippled the medical systems in developing countries but also caused shortages of medical resources in developed countries [8,9]. Hospital visits have plummeted due to fear of COVID-19 [10,11]. According to a report from the Center for Disease Control and Prevention (CDC), in the early stage of the pandemic, the number of emergency patients in the United States dropped by more than 40%, suggesting that many people were reluctant to go to the hospital. Even if they did seek care, hospitals were severely overloaded [12]. All in all, as a large number of COVID-19 patients flooded into the hospitals, patients with other medical conditions were not given the due care, therefore, causing harm to people in a broader sense.

### 2.2. The Containment of the COVID-19 Pandemic

Our study has made contributions to several literature. At first, we provide new evidence that wearing masks can protect people against the COVID-19 pandemic from the perspective of international trade. In previous literature, medical doctors and scholars have pointed out that wearing a mask plays an important role in preventing the spread of COVID-19. Masks protect people around them as well, since the flow resistance of masks effectively prevents the transmission of exhaled air, e.g., when breathing, speaking, singing, coughing, and sneezing [13,14]. Thus, wearing masks reduces the transmissibility per contact by reducing transmission of infected droplets, The reduction of transmission rate could greatly reduce the number of death and economic impact, and the cost of the intervention is very low [15,16]. In Germany, wearing masks has reduced the daily growth rate of reported infections by around 47% [17]. Meanwhile, the WHO advises people to wear masks during the COVID-19 pandemic and provides scientific basis relevant to the use of masks for preventing transmission of COVID-19 [18]. Our study provides cross-country evidence to support the effect of masks.

Then, our study contributes to the literature on China's efforts in fighting the COVID-19 pandemic. Lockdown effectively controls the spread of COVID-19, and the social distancing policies were effective in reducing the impact of the population inflows from the epicentre cities in Hubei Province on the spread of COVID-19 in the destination cities [19]. Stringent quarantines, city lockdowns, and local public health measures imposed in late January, 2020, significantly reduced the spread of the virus [20]. In addition, unprecedented public health efforts in China have contained the spread of this new virus. Measures taken in China are currently proven to reduce human-to-human transmission successfully [21]. China has achieved remarkable results in preventing the spread of the pandemic, ensuring the safety of people's lives, quickly resuming work and production, and promoting economic recovery; in addition, the theoretical framework and successful experience of China's multilevel and multifunctional governance structure are both theoretical and practical and can provide reference for other countries in the world [22]. At the same time, other countries had to stop production because of COVID-19, so the production in China has become the key to providing medical supplies. Taking the pandemic situation in COVID-19 as a natural experiment, this study examines the influence of China's export on other countries' efforts to fight the pandemic situation.

Finally, we have put forward a new perspective on the relationship between international trade and the spread of infectious diseases. In the previous literature, there were some findings about international trade facilitating the spread of the virus. For example, there is a fairly consistent positive relationship between export and new HIV infections. The increase of export will increase the mobility of people (trucking), thus increasing sexual contact [23]. Estimating the impact of export on HIV incidence for sub-Saharan African countries (SSAs), it is found that a doubling per capita export could increase the average HIV incidence by about 55% [24]. Furthermore, the Black plague case originated from foreign merchant ships and then spread to the Asian region along the trade belt [25]. After China's entry into the WTO in 2001, the rapid expansion of international trade promoted the spread of severe acute respiratory syndromes (SARS) in 2003 [26]. On the contrary, we find that when the products traded between countries are antivirus supplies, international trade can help countries around the world overcome difficulties during the pandemic.

## 3. Materials and Methods

The data in this study come from several sources, and the selection and use of these data are explained.

### 3.1. Data Source and Variable Description

#### 3.1.1. Data of COVID-19 Cases

Johns Hopkins University has published the data of COVID-19 cases from all countries in the world (https://coronavirus.jhu.edu/covid-19-daily-video). These data count the development trend of the pandemic in 196 countries and regions in the world including the cumulative number of confirmed, recovered, and deaths per day from January 22, 2020, to now. Meanwhile, this database is still being updated. Since China's customs data are updated to March 2021 and considering the time required for the export and transportation of antivirus supplies and the lag in playing its role, we choose July 31, 2021, to measure the pandemic situation in various countries. After studying existing data and literature, we choose the recovery rate as our important indicator to measure the development degree of the pandemic in various countries. The reasons are as follows.

The number of confirmed cases is an important indicator to measure the severity of a country. However, can we get accurate diagnosis data? For now, this seems unlikely. Calculating coronavirus cases is more difficult than it looks [27]. Scholars find that only considering the number of confirmed cases would be very misleading [28]. One of the characteristics of the COVID-19 is that the infected may be asymptomatic, which will naturally lead to the number of detected cases being less than the actual number. The local detection ability in Africa may also be one of the factors leading to the small number of cases [29].

Although we can obtain death toll of each country in the COVID-19 pandemic, data accuracy is not satisfactory. Since its advent in December 2019, the death toll of COVID-19 has sparked much controversy. Some countries have been reporting the COVID-19 deaths very accurately, while many other countries have been underreporting their COVID-19 deaths by an order of magnitude or more [30]. The official coronavirus death tolls according to Johns Hopkins University are only an estimate. Only countries that have conducted extensive tests can confirm their procedures. Even in those countries that have the necessary medical technologies, the simple act of counting the death toll reflects the chaos caused by COVID-19 [31]. Underestimation caused by insufficient detection and out-of-hospital deaths is an important reason. If you have two concurrent conditions, which classification does it fall to? [32,33]. On the other hand, the influence, review, and manipulation of cases and death data by the top political leaders of some countries could create important impacts on the death toll [33]. For instance, the death toll of coronavirus in the UK is twice that of the official data [34]. Considering these problems, we choose recovery rate as our main explanatory variable to measure the situation of the COVID-19 pandemic in different countries. Although the data of confirmed cases are not satisfactory, it can record the recovered cases more accurately, and the recovery rate is relatively proportional. We divide the number of recovered patients by the number of confirmed cases to express the recovery rate as follows:

(1) $$\begin{array}{c} \text{Recovery}\_{\text{rate}}_{c}=\frac{\text{Recovered }{\text{num}}_{c}}{\text{Confirmed }{\text{num}}_{c}}. \end{array}$$

#### 3.1.2. China's Export of Antivirus Supplies

The data on China's export of antivirus supplies to other countries come from the Chinese Customs Database (https://43.248.49.97/). It contains monthly data of HS8 product from China to 232 countries and regions in the world. By consulting the General Administration of Customs of China and other materials, we have screened out 23 kinds of antivirus supplies, among which 15 kinds are final goods that can be directly used and 8 kinds are intermediate goods used to produce the final goods. The codes and names of these products are given in Table 1; in addition, “final goods = 1” means this product is an end product and “final goods = 0” means this product is an intermediate product.

We have obtained the recovery rate data of various countries and calculated the trade volume and quantity of China's export of antivirus supplies to these countries and regions from January 2018 to March 2020 from China's Customs Database. After merging the above two databases, we get a cross-sectional data of 188 countries.

#### 3.1.3. Other Variables

In order to ensure the unbiasedness of the main coefficients, we sequentially add different control variables to the regression. In this study, the controlled variables from the World Bank's world development indicators include per capita GDP, infant mortality rate, population density, population, and the proportion of people in each country who have completed at least senior high school education. In Section 4.4, we obtained individualism data from different countries from Hofstede insights (https://www.hofstede-insights.com/).

#### 3.1.4. Variable Description

Table 2 provides the basic descriptive statistics of the main variables used in this study. Our main independent variable is the growth rate of China's export of masks or other antivirus supplies. It can be seen from Figure 3 that China's export of antivirus supplies began to increase greatly in April 2020. Therefore, the figure of April 2020 to March 2021 was set up as one year; by comparing it to the data in April 2019 to March 2020, we come up with the export growth rate this year.

At the same time, it can be seen from Figure 2 that the export value of masks dropped sharply after a substantial increase, while the export weight of masks remained at a relatively high level. Considering that this may be influenced by price factors and the amount cannot reflect the real situation of mask export growth, we choose the growth rate of mask export weight as the main explanatory variable.

Figure 4 shows a scatter chart of the growth rate of China's masks weight export and the recovery rate of other countries in the world, which shows the relationship between them intuitively. As shown in Figure 4(a), it is obvious that countries with a higher growth rate of imported masks weight from China have a higher recovery rate. In addition, just as Figure 4(b) suggests, the situation does not always improve when the number of masks increase. There is a peak point, after which the situation does not improve anymore. This means that the demand for masks is nonlinear in the process of fighting the pandemic.

Next, this study uses multiple regression analysis to strictly test the relationship between the growth rate of China's mask export to other countries and the recovery rate of COVID-19 countries.

### 3.2. Empirical Strategy

#### 3.2.1. Regression with Linear Relationship

We explored the linear relationship between the recovery rate and growth rate by the weight of imported masks from China like Figure 4(a). So, we estimate the following linear regression equation:

(2) $$\begin{array}{c} \text{Recovery}\_{\text{rate}}_{c}=\alpha +\beta \;\log\left(\text{increase}\_{\text{rate}}_{c}\right)+\gamma_{i}X_{c}+\varepsilon_{c}. \end{array}$$

In equation (2), the Recovered_rate_*c*_ as the dependent variable refers to the recovery rate of country *c* in the COVID-19 pandemic; log(increase_rate_*c*_) is the logarithm of the growth rate of the country *c*' imports of masks weight from China; *X*_*c*_is a series of control variables, including a series of characteristic values of country *c*; and *ε*_*c*_ is the error term. The OLS method and robust standard errors are used to estimate the model parameters.

The core estimation coefficient is *β* in equation (2), and we expect *β* to be positive. Intuitively, antivirus supplies such as masks will play a role in fighting the pandemic and countries with “panic squeeze of medical resources” imported a lot of antivirus supplies from China which can help them alleviate the shortage of medical resources and improve the recovery rate.

#### 3.2.2. Regression with Nonlinear Relationship

As can be seen from Figure 4(b), there is a nonlinear quadratic relationship between the export of China's masks weight and the recovery rate of various countries in the COVID-19 pandemic. Therefore, we list the following quadratic regression equation and estimate it.

(3) $$\begin{array}{c} \text{Recovery}\_{\text{rate}}_{c}=\alpha +\beta_{1}\text{increase}\_{\text{rate}}_{c}+\beta_{2}\text{increase}\_{\text{rate}}_{c}^{2}+\gamma_{i}X_{c}+\eta_{c}. \end{array}$$

In equation (3), the Recovered_rate*c*_, *X*_*c*_ is consistent with equation (2); increase_rate_*c*_ is the growth rate of the country *c*' imports of masks weight from China; *η*_*c*_ is the error term. As in equation (2), the OLS method and robust standard errors are used to estimate the model parameters.

The core estimation coefficient is *β*_1_ and *β*_2_ in equation (3). We guess *β*_1_ is positive and *β*_2_ is negative. The antivirus supplies such as masks imported from China help countries around the world fight against the COVID-19 pandemic and improve the recovery rate. However, the role of antivirus supplies is not unlimited. When there are enough antivirus supplies, other measures are needed to fight the pandemic.

## 4. Results and Discussion

We removed 8 least-affected countries including Palau and Vatican with less than 100 confirmed cases from the main regression data and added them to the data in Section 4.5.2 for the robustness test.

### 4.1. Linear Effect of Imported Masks

Table 3 provides the main regression results of equation (2). In order to ensure the robustness of the results, we gradually added control variables. From the regression results, it can be seen that the masks imported from China has a positive effect on the fight against the COVID-19 pandemic, and the coefficients are statistically significant.

### 4.2. Nonlinear Effect of Imported Masks

Table 4 provides the main regression results of equation (3). After calculation, the highest point of the quadratic curve is at (10000, 100). There are five countries near and to the right of the point, South Sudan, Sao Tome and Principe, Faroe Islands, Bhutan, and Eritrea. These countries have imported sufficient masks during COVID-19 and thus had better pandemic prevention and control. However, there are more countries to the left of the point with low recovery rate, such as Burundi, Honduras, and Afghanistan. These countries should increase the production and import of masks to combat the pandemic.

### 4.3. The Impact of Different Types of Antivirus Supplies

Our basic results show that masks imported from China increased countries' recovery rates and protected people in countries suffering from the COVID-19 pandemic. In addition to masks, there are many other types of antivirus supplies as given in Table 1. We divide them into final products and intermediate goods according to the different uses. Imported final products can be used directly, such as masks and ventilators. Imported intermediate goods are used to produce final products, such as melt blown cloth and industrial nonautomatic sewing machine.

We separate the import growth of final products and intermediate goods to estimate their respective impacts. The results are given in Table 5 and Table 6. Meanwhile, as shown in Figure 3(a), among all antivirus supplies, the share and growth of the final products occupy a major position, and it also plays an important role in protecting people.

In order to explore the impact of all antivirus supplies, we combine all the commodities given in Table 1 to estimate their total impact.  Table 7 provides this result. Combining the results from Tables 3–7, we find that masks play a pivotal role in fighting the COVID-19 pandemic. During the pandemic, China's export of masks significantly increased the recovery rate in various countries.

### 4.4. The Impact of Collectivism

In 1870, the well-known Hofstede's cultural dimensions theory was proposed, among which individualism and collectivism were important dimensions to measure the cultural differences of different countries. The fundamental problem involved at this level is the degree to which a society keeps interdependence among its members. It has to do with whether people's self-image is defined in terms of “I” or “We.” In individualist societies, people are supposed to take care of themselves and their immediate relatives. In collectivist societies, people belong “in groups” that take care of them in exchange for loyalty. For example, in our data, the United States is the most individualistic country, with an individualism index of 91 (out of 100). In reality, protests against stay-at-home orders broke out in many parts of the United States. Protesters ignored social distancing rules and refused to wear masks [35, 36].

Based on the differences between individualism and collectivism in different countries, we speculate that in countries with strong collectivism, people pay more attention to the combat against COVID-19 for collective safety and importing antivirus supplies plays a greater role.

Therefore, we add the collectivism index as moderating variables to equation (2) and get the following equation.

(4) $$\begin{array}{c} \text{Recovery}\_{\text{rate}}_{c}=\alpha +\rho \left(\text{lgincrease}\_{\text{rate}}_{c}\right)*\left({\text{Mod\_variable}}_{c}\right)+\gamma_{i}X_{c}+\varepsilon_{c}. \end{array}$$

In equation (4), *ρ* is the coefficient we care about most. We performed the centering process of the core explanatory variable and the moderating variables. Then, we multiply the centered variables to get the interaction term. *X*_*c*_ is a series of control variables including the core explanatory variable and the moderating variable. Considering that many countries lack the data of education level, starting from this section, the control variables in the report results do not include education level.

We obtained data from the Hofstede Insights website, which measures the degree of individualism in a country. The higher the indicator value, the stronger the individualism of the country. We use 100 minus level of individualism as the level of collectivism. We put this variable as a moderating variable into the regression and the results are given in Table 8.

This result confirms our speculation that in countries with stronger collectivism, imported antivirus supplies play a greater role in protecting people. At the same time, although only the results of total amount of antivirus supplies show statistically significant results, we think this conclusion is effective due to the lack of data on collectivism indicators.

### 4.5. Additional Robustness Check

#### 4.5.1. Change the Calculation Data of Growth Rate

In the previous regression, our explanatory variable is the growth rate of masks, which is the growth rate of imports from April 2020 to March 2021 compared to April 2019 to March 2020. In this section, we change the data to the growth rate of China and use the growth rate in 2020 compared to 2019 as the main independent variable.

Table 9 provides our results, which are consistent with the basic regression results. Considering the lack of data on education levels of each country, the control variables in the results reported in this section only include GDP per capita, infant mortality, population density, and population level. This result is consistent with our main results.

#### 4.5.2. Use Complete Sample

In the regression of the main result, we removed eight countries that are less affected by the COVID-19 pandemic, which had fewer than 100 confirmed cases as of July 31, 2021. In this section, we include these countries again in the data for robustness testing. We use cross-sectional data for 188 countries to estimate the regression equation.

The estimated results are given in Table 10. As in Section 6.1, the control variables in the results reported in this section include only GDP per capita, infant mortality, population density, and population level. This result again supports our findings.

### 4.6. Discussion

Compared with exiting literature on international trade and the spread of virus, different from previous research that international trade promotes the spread of the virus, our findings support the significant role of masks' export in fighting against the COVID-19 pandemic. We also explore the impact of final goods, intermediate goods, and total antivirus supplies on the recovery rate of each country. We find that these effects are not significant and masks play a pivotal role in fighting the COVID-19 pandemic.

To explore the role of collectivism in this relationship, we add the collectivism index to our regression. This result shows that in countries with stronger collectivism, imported antivirus supplies play a greater role in protecting people and we think this conclusion is effective due to the lack of data on collectivism indicators.

Then, in order to investigate the robustness of the results, we conduct robustness tests through changing the calculation data of growth rate and using complete sample. These results all confirm the credibility of the results of this study.

## 5. Conclusions

Since the outbreak of COVID-19 at the end of 2019, the pandemic has not been completely controlled yet. The COVID-19 pandemic has a wide range of influence, and it has brought great harm to public health around the world. In this study, the influence of China's masks on the recovery rate of various countries is investigated by using cross-border data. We find that China's masks have a positive impact on countries around the world in fighting the pandemic. Our findings may have some policy implications.

First, wearing a mask plays an important role in preventing COVID-19 pandemic, which are confirmed by many medical research, while our findings provide new evidence from the perspective of international trade. Second, this study supplements the existing literature, and international trade may not only facilitate the spread of the virus. When the traded products are antivirus supplies, international trade will play a positive role in pandemic containment. Third, after the outbreak of the pandemic, China has achieved good results through its unremitting efforts, and the pandemic has been effectively controlled [19–22], which provides valuable lessons for the countries still in dire straits. Meanwhile, China's rapid resumption of production and exports of antivirus supplies have both played a pivotal role in the fight against COVID-19 globally.

It is worth noting that confirmed and mortality statistics are fundamental to public health decision making. However, as introduced in Section 3.1.1, there is currently no cross-country comparable statistics on the number of confirmed and death cases. This impedes us to investigate the trade of masks on the confirmed rate, fatality rate, or mortality rate, which are more important. Further research needs the support of more accurate and scientific databases of COVID-19 cases.

## Figures and Tables

**Figure 1:** (a) The cumulative confirmed/recovered/death cases of COVID-19 in the world. (b) The newly confirmed/recovered/death cases of COVID-19 in the world.

**Figure 2:** China's exports of antivirus supplies and the world's total exports.

**Figure 3:** (a) China's monthly export value of antivirus supplies. (b) China's monthly export value and weight of masks.

**Figure 4:** (a) The linear relationship between China's export growth rate of mask weight and recovery rate of countries. (b) The nonlinear relationship between China's export growth rate of mask weight and recovery rate of countries.

**Table 1:** HS8 code and name of antivirus supplies.

HS8	Name	Final goods = 1
22071000	Medical alcohol in nonretail packaging, >80%	1
22089090	Medical alcohol in nonretail packaging, <80%	1
38089400	Medical alcohol and retail packaging medical alcohol 75%	1
39262011	Protective gloves (plastic PVC)	1
39262019	Protective gloves (plastic other)	1
39262090	Medical protective clothing (plastic)	1
40151100	Protective gloves (for rubber surgery)	1
40151900	Protective gloves (rubber others)	1
40159010	Medical protective clothing (rubber)	1
56031190	Nonwoven fabrics made of other chemical fiber filaments (melt blown cloth)	0
56031290	Nonwoven fabrics made of other chemical fiber filaments (melt blown cloth)	0
62101030	Medical protective clothing (chemical fiber), surgical clothing	1
63079000	Ordinary medical masks and medical surgical masks	1
84201000	Seam sealing machine	0
84522900	Industrial nonautomatic sewing machine	0
84490090	Flat mask production equipment, cup-shaped mask production equipment, and folding mask production equipment	0
90049090	Goggles	1
90181930	Patient monitor	1
90192000	Ventilator (ozone therapy machine and oxygen therapy machine)	1
90251990	Infrared thermometer	1
39269090	Plastic nose clip	0
90259000	Infrared thermometer sensor element	0
65061000	Mask airtightness test airtight cover	0

**Table 2:** Descriptive statistics of each variable.

Variable	Variable explanation	Obs.	Mean	SD	Min	Max
Recovery rate	Recovery rate of COVID-19 cases	188	85.0853	19.6513	0	100
Log (increase rate)	Logarithm of the China's masks weight imported by various countries	188	5.8492	1.0293	3.1664	9.9170
Increase rate	Growth rate of China's masks weight imported by various countries	188	720.8164	2279.54	−76.2791	20172.34
Increase rate^2^	The square of the weight growth rate of masks imported from China by various countries	188	5688238	3.79e + 07	22.2552	4.07e + 08
Log (per GDP)	Logarithm of the GDP per capita	183	8.7562	1.4745	5.5655	12.1575
Infant mortality	Infant mortality in each country	184	21.2544	19.4605	1.5	81
Log (population density)	Logarithm of the population density	187	4.3185	1.4865	−1.9879	9.8639
Log (population)	Logarithm of the population	188	15.5836	2.2430	6.6859	21.0355
Education level	Percentage of at least completed high school education	120	51.8516	26.8309	2.8055	97.3998
Collectivism	Collectivism index = 100−individualism index	106	62.5943	20.8230	9	94

**Table 3:** The linear impact of mask imports.

Recovery rate	(1)	(2)	(3)	(4)	(5)	(6)
Log (increase rate)	2.974^*∗∗∗*^	2.898^*∗∗∗*^	3.113^*∗∗∗*^	3.137^*∗∗∗*^	2.917^*∗∗∗*^	3.768^*∗∗∗*^
	(1.039)	(1.191)	(1.291)	(1.308)	(1.337)	(1.890)
Log (per GDP)		2.915^*∗∗∗*^	2.805	2.815	2.486	1.249
		(0.983)	(1.761)	(1.775)	(1.831)	(2.273)
Infant mortality			−0.006	−0.008	−0.019	0.106
			(0.118)	(0.116)	(0.118)	(0.207)
Log (population density)				−0.262	−0.320	0.172
				3.137^*∗∗∗*^	(0.811)	(1.163)
Log (population)					−0.632	−0.201
					(0.563)	(0.854)
Education level						0.139^*∗*^
						(0.081)
Obs.	180	176	173	173	173	114
R-squared	0.029	0.086	0.082	0.083	0.087	0.075

^*∗*^Significant at 10%. ^*∗∗∗*^Significant at 5%. ^*∗∗∗*^Significant at 1%.

**Table 4:** The nonlinear impact of mask imports.

Recovery rate	(1)	(2)	(3)	(4)	(5)	(6)
Increase rate	0.003^*∗∗∗*^	0.004^*∗∗∗*^	0.004^*∗∗∗*^	0.005^*∗∗∗*^	0.004^*∗∗∗*^	0.005^*∗∗∗*^
	(0.001)	(0.001)	(0.002)	(0.002)	(0.002)	(0.002)
Increase rate^2^	−0.000^*∗∗∗*^	−0.000^*∗∗∗*^	−0.000^*∗∗∗*^	−0.000^*∗∗∗*^	−0.000^*∗∗∗*^	−0.000^*∗∗∗*^
	(0.000)	(0.000)	(0.000)	(0.000)	(0.000)	(0.000)
Log (per GDP)		3.060^*∗∗∗*^	3.047^*∗*^	3.055^*∗*^	2.726	1.429
		(1.004)	(1.784)	(1.797)	(1.860)	(2.324)
Infant mortality			−0.006	−0.009	−0.019	0.084
			(0.118)	(0.116)	(0.118)	(0.211)
Log (population density)				−0.223	−0.285	0.369
				(0.803)	(0.813)	(1.179)
Log (population)					−0.590	−0.140
					(0.572)	(0.858)
Education level						0.135^*∗*^
						(0.080)
Obs.	180	176	173	173	173	114
R-squared	0.022	0.086	0.085	0.085	0.088	0.074

^*∗*^Significant at 10%. ^*∗∗∗*^Significant at 5%. ^*∗∗∗*^Significant at 1%.

**Table 5:** The impact of final goods.

Recovery rate	(1)	(2)	(3)	(4)	(5)	(6)
Linear impact of final goods						
Log (increase rate)	1.878^*∗*^	1.662	1.969	2.052	1.702	1.683
	(1.055)	(1.136)	(1.358)	(1.376)	(1.397)	(1.937)
Log (per GDP)		2.908^*∗∗∗*^	2.501	2.498	2.263	1.186
		(1.022)	(1.858)	(1.858)	(1.882)	(2.461)
Infant mortality			−0.028	−0.033	−0.039	0.107
			(0.121)	(0.120)	(0.121)	(0.212)
Log (population density)				−0.370	−0.393	−0.020
				(0.811)	(0.816)	(1.169)
Log (population)					−0.584	−0.269
					(0.539)	(0.806)
Education level						0.122
						(0.079)
Obs.	180	176	173	173	173	114
R-squared	0.015	0.074	0.070	0.071	0.074	0.047

Nonlinear impact of final goods						

Increase rate	0.001	0.001	0.003^*∗*^	0.003^*∗*^	0.002	0.001
	(0.001)	(0.001)	(0.001)	(0.001)	(0.002)	(0.004)
Increase rate^2^	−0.000	−0.000	−0.000^*∗*^	−0.000^*∗*^	−0.000	0.000
	(0.000)	(0.000)	(0.000)	(0.000)	(0.000)	(0.000)
Log (per GDP)		3.071^*∗∗∗*^	2.630	2.636	2.407	1.555
		(1.028)	(1.822)	(1.829)	(1.858)	(2.595)
Infant mortality			−0.030	−0.035	−0.039	0.130
			(0.121)	(0.119)	(0.120)	(0.217)
Log (population density)				−0.367	−0.390	0.095
				(0.805)	(0.811)	(1.135)
Log (population)					−0.514	−0.202
					(0.598)	(0.865)
Education level						0.129
						(0.080)
Obs.	180	176	173	173	173	114
R-squared	0.011	0.073	0.074	0.075	0.077	0.052

^*∗*^Significant at 10%. ^*∗∗∗*^Significant at 5%. ^*∗∗∗*^Significant at 1%.

**Table 6:** The impact of intermediate goods.

Recovery rate	(1)	(2)	(3)	(4)	(5)	(6)
Linear impact of intermediate goods						
Log (increase rate)	1.823	1.873	1.790	1.778	1.566	2.718
	(1.431)	(1.466)	(1.625)	(1.621)	(1.606)	(3.188)
Log (per GDP)		3.365^*∗∗∗*^	3.670^*∗*^	3.670^*∗*^	3.313^*∗*^	1.968
		(1.069)	(1.914)	(1.923)	(1.955)	(2.574)
Infant mortality			0.030	0.032	0.022	0.135
			(0.124)	(0.122)	(0.123)	(0.213)
Log (population density)				0.146	0.065	0.829
				(0.801)	(0.817)	(1.263)
Log (population)					−0.711	0.125
					(0.575)	(0.907)
Education level						0.144
						(0.094)
Obs.	168	165	163	163	163	106
R-squared	0.008	0.081	0.077	0.077	0.082	0.065

Nonlinear impact of intermediate goods						

Recovery rate	(1)	(2)	(3)	(4)	(5)	(6)
Increase rate	0.012	0.012	0.013	0.014	0.011	0.009
	(0.011)	(0.011)	(0.012)	(0.012)	(0.012)	(0.068)
Increase rate^2^	−0.000	−0.000	−0.000	−0.000	−0.000	−0.000
	(0.000)	(0.000)	(0.000)	(0.000)	(0.000)	(0.000)
Log (per GDP)		3.212^*∗∗∗*^	2.683	2.689	2.322	1.442
		(1.032)	(1.827)	(1.845)	(1.872)	(2.142)
Infant mortality			−0.047	−0.048	−0.057	0.133
			(0.123)	(0.121)	(0.123)	(0.212)
Log (population density)				−0.144	−0.210	0.196
				(0.788)	(0.797)	(1.075)
Log (population)					−0.730	−0.610
					0.011	(1.001)
Education level						0.117
						(0.080)
Obs.	180	176	173	173	173	114
R-squared	0.007	0.076	0.072	0.072	0.077	0.041

^*∗*^Significant at 10%. ^*∗∗∗*^Significant at 5%. ^*∗∗∗*^Significant at 1%.

**Table 7:** The impact of total antivirus supplies.

Recovery rate	(1)	(2)	(3)	(4)	(5)	(6)
Linear impact of total virus supplies						
Log (increase rate)	2.936^*∗∗∗*^	2.151	2.319	2.380	2.005	1.908
	(1.392)	(1.478)	(1.644)	(1.633)	(1.681)	(2.828)
Log (per GDP)		2.741^*∗∗∗*^	2.332	2.329	2.110	1.034
		(1.057)	(1.946)	(1.945)	(1.955)	(2.711)
Infant mortality			−0.031	−0.035	−0.040	0.107
			(0.123)	(0.121)	(0.122)	(0.214)
Log (population density)				−0.317	−0.352	0.039
				(0.797)	(0.804)	(1.159)
Log (population)					−0.593	−0.277
					(0.552)	(0.804)
Education level						0.121
						1.908
Obs.	178	175	173	173	173	114
R-squared	0.025	0.074	0.071	0.072	0.075	0.046

Nonlinear impact of total antivirus supplies						

Increase rate	0.007^*∗∗∗*^	0.005	0.006	0.014	0.006	0.004
	(0.003)	(0.003)	(0.004)	(0.012)	(0.004)	(0.013)
Increase rate^2^	−0.000^*∗∗∗*^	−0.000	−0.000	−0.000	−0.000	−0.000
	(0.000)	(0.000)	(0.000)	(0.000)	(0.000)	(0.000)
Log (per GDP)		2.891^*∗∗∗*^	2.483	2.689	2.486	1.264
		(1.044)	(1.901)	(1.845)	(1.906)	(2.860)
Infant mortality			−0.031	−0.048	−0.034	0.116
			(0.121)	(0.121)	(0.119)	(0.223)
Log (population density)				−0.144	−0.294	0.079
				(0.788)	(0.792)	(1.142)
Log (population)					0.006	−0.334
					(0.004)	(0.859)
Education level						0.120
						(0.080)
Obs.	180	176	173	173	173	114
R-squared	0.021	0.075	0.071	0.072	0.071	0.043

^*∗*^Significant at 10%. ^*∗∗∗*^Significant at 5%. ^*∗∗∗*^Significant at 1%.

**Table 8:** The impact of collectivism.

Recovery rate	Masks' weight	Final goods	Intermediate goods	Total supplies
Log (increase rate)^*∗*^collectivism	0.160 (0.118)	0.189 (0.130)	0.190 (0.158)	0.320^*∗∗∗*^ (0.149)
Control variables	YES	YES	YES	YES
Obs.	104	104	101	104
R-squared	0.062	0.070	0.054	0.102

^*∗*^Significant at 10%. ^*∗∗∗*^Significant at 5%. ^*∗∗∗*^Significant at 1%.

**Table 9:** Change the calculation data of growth rate.

Recovery rate	Masks' weight		Final goods		Intermediate goods		Total supplies	
	Nonlinear	Linear	Nonlinear	Linear	Nonlinear	Linear	Nonlinear	Linear
Increase rate	0.006^*∗∗∗*^		0.004^*∗*^		0.013		0.004	
	(0.002)		(0.002)		(0.010)		(0.003)	
Increase rate^2^	−0.000^*∗∗∗*^		−0.000^*∗*^		−0.000		−0.000	
	(0.000)		(0.000)		(0.000)		(0.000)	
Log (increase rate)		5.230^*∗∗∗*^		2.580		1.637		2.598
		(2.003)		(1.604)		(1.464)		(1.921)
Control variables	YES	YES	YES	YES	YES	YES	YES	YES
Obs.	180	180	180	180	180	169	173	173
R-squared	0.079	0.104	0.064	0.059	0.085	0.085	0.076	0.076

^*∗*^Significant at 10%. ^*∗∗∗*^Significant at 5%. ^*∗∗∗*^Significant at 1%.

**Table 10:** Use complete sample.

Recovery rate	Masks' weight		Final goods		Intermediate goods		Total supplies	
	Nonlinear	Linear	Nonlinear	Linear	Nonlinear	Linear	Nonlinear	Linear
Increase rate	0.004^*∗∗∗*^		0.001^*∗*^		−0.002		0.009^*∗*^	
	(0.001)		(0.001)		(0.028)		(0.005)	
Increase rate^2^	−0.000^*∗∗∗*^		−0.000^*∗*^		0.000		−0.000	
	(0.000)		(0.000)		(0.000)		(0.000)	
Log (increase rate)		2.950^*∗∗∗*^		1.991		1.158		4.041^*∗*^
		(1.304)		(1.292)		(3.374)		(2.379)
Control variables	YES	YES	YES	YES	YES	YES	YES	YES
Obs.	173	173	173	173	173	173	180	180
R-squared	0.085	0.087	0.076	0.076	0.069	0.067	0.064	0.078

^*∗*^Significant at 10%. ^*∗∗∗*^Significant at 5%. ^*∗∗∗*^Significant at 1%.

## Data Availability

The data used to support this study are from publicly available datasets and are available from the corresponding author upon request.
